# Integrated Bioinformatics Analysis for Identification of the Hub Genes Linked with Prognosis of Ovarian Cancer Patients

**DOI:** 10.1155/2022/5113447

**Published:** 2022-01-10

**Authors:** Xiaofeng Li, Qiu Wang, Zhicheng Wu, Jiantong Zheng, Ling Ji

**Affiliations:** ^1^Department of Laboratory Medicine, Peking University Shenzhen Hospital, Shenzhen, China; ^2^Shenzhen Dymind Biotechnology Company Limited, China

## Abstract

**Background:**

One of the most usual gynecological state of tumor is ovarian cancer and is a major reason of gynecological tumor-related global mortality rate. There have been multiple risk elements related to ovarian cancer like the background of past cases associated with breast cancer or ovarian cancer, or excessive body weight issues, case history of smoking, and untimely menstruation or menopause. Because of unclear expressions, more than 70% of the ovarian cancer patient cases are determined during the early stage. *Material and Methods.* GSE38666, GSE40595, and GSE66957 were the three microarray datasets which were analyzed using GEO2R for screening the differentially expressed genes. GO, Kyoto Encyclopedia of Genes, and protein expression studies were performed for analysis of hub genes. Then, survival analysis was performed for all the hub genes.

**Results:**

From the dataset, a total of 199 differentially expressed genes (DEGs) were identified. Through the KEGG pathway study, it was noted that the DEGs are mainly linked with the AGE-RAGE signaling pathway, central carbon metabolism, and human papillomavirus infection. The survival analysis showed 4 highly expressed hub genes COL4A1, SDC1, CDKN2A, and TOP2A which correlated with overall survival in ovarian cancer patients. Moreover, the expression of the 4 hub genes was validated by the GEPIA database and the Human Protein Atlas.

**Conclusion:**

The results have shown that all 4 hub genes were found to be upregulated in ovarian cancer tissues which predict poor prognosis in patients with ovarian cancer.

## 1. Introduction

Ovarian cancer is a usual gynecological state of a malignant tumor that leads to gynecological cancer-associated global mortality rate [1, 2]. There is an approximate count of 250,000 fresh cases where 160,000 death cases were reported in 2018 [3]. There are numerous components encompassing a family background of ovarian cancer which involves smoking, untimely menstruation, or even overdue menopause and infertility in birth that are proposed to promote the spread of ovarian cancer [4]. The prime remedy scheme for the ovarian cancer involves surgical process of resection along with chemotherapy. Though, around more than 50% of the cases from ovarian cancer are identified at an overdue period, as the productive diagnosis for the case of ovarian cancer is still restrained [5].

The approach of gene expression is considered to be a powerful procedure which is constructed on a differentially expressed genes (DEGs) and can be shielded in between the suffering as well as the healthy people [6]. The differentially expressed genes can be utilized to investigate the molecular signal pathways in order to examine the gene managing system in multiple disorders which comprises of epithelial ovarian cancer (EOC). In the present time, various differentially expressed genes have been discovered which may be comprised in the formation as well as the advancement of ovarian cancer [7], but the outcomes are unpredictable because of varying tissues, dimensions of the sample, and the varied bioinformatics analysis procedures and the platforms for observation. The investigation of independent experiment involves high uncertainty of bias, along with consolidated analysis of different databases which could enhance the characteristics and the definitiveness of the identification of differentially expressed genes.

The growing count of procedures involved in bioinformatics has been utilized to discover the prognostic biomarkers in the neoplastic disorders, although the overall survival (OS) of the rate of people suffering with ovarian cancer lasts below par. The evaluation of microarray-based gene expression is one of the most frequently utilized high-throughput and thriving approaches which is used to analyze the complex disease pathogenesis [8]. Although the researches which were carried out used human ovarian cancer gene expression profiling were rarely found, there have been technologies formed which yield high-throughput so as to determine new biomarkers and therapeutic targets in various types of cancers incorporating the ovarian cancer [9–11].

Additionally, varied researches have examined the Gene Expression Omnibus (GEO) collections of related datas and determined hub genes affiliated with the prognosis of ovarian cancer [8, 12]. There is further investigation of the Gene Expression Omnibus datasets by utilizing different methods which can help in investigating the biomarkers and the primary process responsible for development of ovarian cancers and to issue new awareness into the present study in the ovarian cancer.

## 2. Material and Methods

The GEO database (https://www.ncbi.nlm.nih.gov/gds) was used for downloading microarray dataset which is an open repository. Three datasets were downloaded GSE38666, GSE40595, and GSE66957 for analysis. The research procedure is indicated in Figure 1.

### 2.1. Enrichment Pathway and Functional Analysis

Enrichment analysis for Gene Ontology and KEGG pathway was done using online program (xiantao: https://www.xiantao.love/), which was built based on R. *P* < 0.05 is the cutoff criteria.

### 2.2. Differentially Expressed Gene (DEG) Selection

DEG processing used the GEO2R tool (http://www.ncbi.nlm.nih.gov/geo/geo2r/). |log2 fold change| > 1.5 and *P* < 0.05 were set at the cutoff values.

### 2.3. PPI Network and Module Analyses

The STRING database (http://string-db.org) was composed of upregulated and downregulated DEGs that was built, with a cutoff score more than 0.4. Using the clusterone add-in of Cytoscape v3.9.0 to pick the significant modules from the PPI network (https://cytoscape.org/) with *P* < 0.01 showed statistical importance. The degree was executed by two add-ins CentiScaPe and Molecular Complex Detection (MCODE) in Cytoscape to illuminate the modules and most significant nodes in the network.

### 2.4. Validation and Expression of Hub Gene in Ovarian Cancer

The expression levels of hub genes are shown in GEPIA (based on TCGA data) (http://gepia.cancer-pku.cn). *P* < 0.05 was viewed to show a statistically important difference in these analyses.

### 2.5. Survival Analysis

The survival analysis of DEGs was performed using the Kaplan–Meier plotter (KM plotter, http://www.kmplot.com). The hazard ratio (HR) with 95% confidence intervals and log-rank *P* value were calculated and displayed on the webpage.

### 2.6. Expression Analysis

The expressions of the hub genes were further confirmed in the GEPIA database. The protein expression of the hub genes was validated in the Human Protein Atlas (http://www.proteinatlas.org/).

### 2.7. Availability of Data and Materials

The datasets analyzed for this study can be found in the GEO datasets (https://www.ncbi.nlm.nih.gov/gds), TCGA database, and the Human Protein Atlas.

## 3. Results

### 3.1. DEG Screening and Analysis

We used the GEO2R tool to analyze the DEGs, and the DEGs were shown using volcano plots (Figures 2(a)–2(c)). A total of 4033, 822, and 6095 genes were identified in the GSE38666, GSE40595, and GSE66957, respectively. A total of 199 common DEGs were identified by using the Venn diagram (Figure 2(d)).

### 3.2. GO and KEGG Enrichment Analysis

A total of 199 genes were identified by enrichment analysis, with *P* (by less than 0.05) statistical significance used to be determined.  Figure 2 displays GO-BP, CC, MF, and KEGG pathway results. The top 3 GO terms are significantly enriched in “extracellular structure organization,” “extracellular matrix organization,” “epithelial tube morphogenesis,” “extracellular matrix component,” “collagen trimer,” “collagen-containing extracellular matrix,” “platelet-derived growth factor binding,” “extracellular matrix structural constituent conferring tensile strength,” and “extracellular matrix structural constituent.” The KEGG pathways of DEGs were primarily enriched in “human papillomavirus infection,” “central carbon metabolism in cancer,” and “AGE-RAGE signaling pathway in diabetic complications” (Figure 3).

### 3.3. Protein Interaction Network and Hub Gene Analysis

To study common genes' relationship between modules, protein interaction networks were built by using Cytoscape software (V3.9.0) that was based on the STRING database results (Figure 4(a)). Further, the *k*-core analysis was executed to discover the hub genes and cardinal clusters of PPI networks. By Cytoscape-MCODE analysis, by using the cytoHubba module, the top 20 genes with the highest scores were identified from the PPI network (Figure 4(b)). At last, the genes that were identified both in cytoHubba and MCODE analysis were defined by hub genes, and a total of 18 hub genes were chosen for further survival analysis.

### 3.4. Survival Analysis of Hub Genes

The overall survival rate (OS) role of hub genes in ovarian cancer was analyzed by the online database (https://kmplot.com/analysis/index.php?p=service). As shown in Figure 5, 1,656 ovarian cancer patients were contained in the OS analysis. We found high expression of COL4A1 (Figure 5(a)), SDC1 (Figure 5(b)), CDKN2A (Figure 5(c)), and TOP2A (Figure 5(d)) significantly associated with shorter OS of the patients with ovarian cancer. However, the other hub genes had no significant association with OS of the patients (data not shown).

### 3.5. Expression of Hub Gene in Ovarian Cancer

We used TCGA data of ovarian cancer to validate the four hub gene expression with the online tool of GEPIA. All of the four hub genes are expressed differently in cancer and normal tissues of the ovary by the criterion of |logFC| > 1 and *P* < 0.01 (Figure 6). Moreover, the protein expression of hub genes including COL4A1 (Figure 7(a)), CDKN2A (Figure 7(b)), SDC1 (Figure 7(c)), and TOP2A (Figure 7(d)) was analyzed by using the Human Protein Atlas, and the protein expression levels of these genes were significantly higher in the ovarian cancer tissues than that in the normal ovarian tissues.

## 4. Discussion

A lot of researches have been established for ovarian cancer where the prognosis of patients is still very poor. Therefore, for identification of potential biomarkers, a lot of detailed study including treatment options, pathways, mechanisms, and prognosis has to be studied [13–15]. Recent growth in bioinformatical analysis sector includes data sequencing, microarray analysis, bioinformatical analysis, and studying of genetic alterations for understating the pathophysiology of ovarian cancer [16–18]. In this study, we have analyzed differentially expressed genes from three GEO datasets (GSE38666, GSE40595, and GSE66957). It was found that 199 common DEG regulated genes. Further analysis of GO and KEGG pathways were also performed.

The KEGG pathway has shown that the differentially expressed gene was mostly related to the “human papillomavirus infection,” “central carbon metabolism in cancer,” and “AGE-RAGE signaling pathway in diabetic complications.” Also, the results have given clear idea that analysis of molecular interactions is insightful in case of ovarian cancer. Further studies on survival analysis were done where four hub genes were highly expressed COL4A1, SDC1, CDKN2A, and TOP2A. These were showing correlation with ovarian cancer patients. The dysregulation of these hub genes are linked with the genesis and progression of ovarian cancer.

Collagen IV is the most abundant constituents of basement membranes of ECM [19]; COL4A1 encode collagen IV alpha 1 chain, together with COL4A2 to assemble into *α*1*α*1*α*2 heterodimers (Col IV), then secreted into extracellular matrix [20]. Increased COL4A1 promotes tumor invasion via induction of tumor budding in bladder cancer cells [21]. Upregulated COL4A1 contributes to the proliferation and migration of breast cancer cells [22]. However, the detailed mechanisms of COL4A1 in ovarian cancer have not been elucidated.

Overexpression of SDC1 in many types of cancers contributes to cell proliferation, cell migration, and cell-matrix interactions via its receptor for extracellular matrix proteins [23–25]. In case of ovarian cancer, SDC1 promotes the adhesion and migration of epithelial cells. Thus, SDC1 promotes the transformation in malignancy of ovarian cancer [26, 27]. Our results have also shown that upregulated SDC1 in the tissues of ovarian cancer and increased expression of SDC1 are correlational to the bad prognosis in patients of ovarian cancer which was analyzed by our bioinformatical study.

The role of TOP2A is to encode DNA topoisomerase [28]; it also plays a strong role in regulation of transcription, replication, and repair of DNA [29, 30]. A lot of studies also suggest that involvement of carcinogenesis in various cancers (lung, liver, and breast cancer) is due to highly expressed TOP2A thereby causing slow prognosis in patients [31–33]. TOP2A also promotes tumorigenesis in ovarian cancer which regulates the TGF-*β*/Smad pathway; the expression of TOP2A was also found to correlate with poor survival of ovarian cancer patients and platinum resistance [34, 35]. Our results have shown that upregulation of TOP2A in tissues of ovarian cancer is linked with poor prognosis.

The current study shows that a total of 199 DEGs were identified in our integrated bioinformatical analysis. A total of 4 hub genes, namely, COL4A1, SDC1, CDKN2A, and TOP2A were found to be upregulated in ovarian cancer tissues which were also responsible for the poor prognosis in patients. More studies must be performed for investigating the mechanism of all these hub genes in ovarian cancer.

## Figures and Tables

**Figure 1:** The study procedure.

**Figure 2:** Identification of common DEGs. Volcano plots of DEGs in (a) GSE38666, (b) GSE40595, and (c) GSE66957 are shown. (d) Venn diagram shows the common DEGs in the datasets.

**Figure 3:** GO and KEGG results of DEGs. GO: Gene Ontology; KEGG: Kyoto Encyclopedia of Genes and Genomes.

**Figure 4:** PPI network and module analysis of DEGs. (a) PPI network of DEGs obtained from the STRING database. (b) Submodule network analyzed by cytoHubba, and top 20 genes are shown.

**Figure 5:** The correlation analysis between hub genes and OS of ovarian cancer patients. The association between the expression levels of (a) COL4A1, (b) SDC1, (c) CDKN2A, and (d) TOP2A and the OS of ovarian cancer patients was analyzed by the KM plotter. Abbreviation: HR: hazard ratio.

**Figure 6:** The transcriptional differences of hub gene levels between ovarian cancer tissues and normal tissues in TCGA.

**Figure 7:** Analysis of protein expression of four hub genes. The protein expression of (a) COL4A1, (b) CDKN2A, (c) SDC1, and (d) TOP2A in normal ovarian tissues and ovarian cancer tissues was obtained from the Human Protein Atlas.

## Data Availability

The data used to support this study are available from the corresponding author upon request.
